# Classification System of National Music Rhythm Spectrogram Based on Biological Neural Network

**DOI:** 10.1155/2022/2047576

**Published:** 2022-10-12

**Authors:** Dan Mi, Lu Qin

**Affiliations:** ^1^Department of Music, Xinxiang University, Xinxiang, Henan 453003, China; ^2^Department of Sports, Xinxiang University, Xinxiang, Henan 453003, China

## Abstract

National music is a treasure of Chinese traditional culture. It contains the cultural characteristics of various regions and reflects the core value of Chinese traditional culture. Classification technology classifies a large number of unorganized drama documents, which are not labeled, and to some extent, it helps folk music better enter the lives of ordinary people. Simulate folk music of different spectrum and record corresponding music audio under laboratory conditions Through Fourier transform and other methods, music audio is converted into spectrogram, and a total of 2608 two-dimensional spectrogram images are obtained as datasets. The sonogram dataset is imported into the deep convolution neural network GoogLeNet for music type recognition, and the test accuracy is 99.6%. In addition, the parallel GoogLeNet technology based on inverse autoregressive flow is used. The unique improvement is that acoustic features can be quickly converted into corresponding speech time-domain waveforms, reaching the real-time level, improving the efficiency of model training and loading, and outputting speech with higher naturalness. In order to further prove the reliability of the experimental results, the spectrogram datasets are imported into Resnet18 and Shufflenet for training, and the test accuracy of 99.2% is obtained. The results show that this method can effectively classify and recognize music. The experimental results show that this scheme can achieve more accurate classification. The research realizes the recognition of national music through deep learning spectrogram classification for the first time, which is an intelligent and fast new method of classification and recognition.

## 1. Introduction

Music classification is an important part of multimedia applications. With the rapid development of data storage, compression technology, and Internet technology, music type data have increased dramatically. Traditional manual retrieval methods can no longer meet the needs of massive music information retrieval and classification. The computer automatic classification of music is to solve the above problems. The computer automatic recognition of music is a new interdisciplinary subject. Its research involves physics, signal processing, human-computer interaction, music theory, music psychology, and many other disciplines. Its main task is to obtain the relevant information of music content through the processing and feature extraction of audio signals, which can be used for comparison, classification, and even automatic recording [1]. Therefore, it is urgent to adopt new technologies to effectively manage massive music resources. However, this method requires manual annotation of massive databases, and the workload is very huge. Another method is to manage according to the content of music, that is, index and retrieve from the music database according to the rhythm, sound quality, and melody characteristics of music [2].

Music classification is essentially a problem of pattern recognition, which mainly includes two aspects: feature extraction and classification. Many researchers have done a lot of work in this field. Using univariate autoregressive integrated moving average (ARIMA) model and nonlinear autoregressive exogenous (NARX) model to classify music, the average absolute error and mean square error of the database are 5.5% and 10.6%, respectively. The average absolute error and mean square error of 10 min database are 2.3% and 12.8%, respectively. The support vector machine (SVM) is adopted to music classification and has achieved high prediction accuracy and convergence speed. Based on the modeling technology of chaotic time series and the wind music classification strategy of Apriori algorithm, the chaotic characteristics of music rhythm time series are analyzed, and its significance to music classification is discussed [3]. Literature [4] classifies music using a double-layer emotional classification model based on AdaBoost. The paper points out that the first layer of the system classifies according to the intensity and time-domain characteristics of music signals, and the second layer classifies according to the rhythmic characteristics of music signals. Finally, according to the classification results of the two-level classifiers and the weights of each level of classifiers, the final classification results are obtained by matching and accumulating. Literature [5] attributes the spectrum classification of music to the problem of regression. According to quality, melody, and rhythm characteristics of music, SVR regression algorithm is used to calculate the arousal and value values of each song and locate them in the emotion plane proposed by Thayer. Search the music songs you need according to the explicit values of arousal and valance. Literature [6] proposed using BP neural network algorithm to classify MIDI music files. Literature [7] uses GMM machine learning algorithm to detect and track music emotion. Siphocly and others [8] proposed a double-layer SVM model for music emotion classification. It can be seen that the classification of music emotion has been fully concerned by the academic community [9].

Since its birth, deep learning has been favored by many researchers. It has been widely used in many fields, such as food detection [10], medical detection [11], face recognition [12], emotion recognition [13], crop recognition [14], image enhancement [15], and machine control [16], and researchers have also begun to apply it to the field of music classification and recognition. Literature [16] uses neural network to predict the uncertain input data expressed in the form of interval. The purpose is to quantify the uncertainty generated by the input data and prediction model in the prediction and finally train a high-performance multilayer perceptron neural network, so as to realize the classification of music. Literature [17] uses deep learning self-encoder for short-term music prediction. The proposed CNN model is superior to the classical DNN model and the DNN model with shallow structure. Literature [18] predicts music based on time series prediction and extreme value optimization. Based on empirical wavelet transform, long-term and short-term memory neural network, Elman neural network and other deep learning methods for music type recognition, the results show that the model has good performance in high-precision music recognition [20, 21]. Although more and more researchers are aware of the importance of deep learning technology in the field of music type recognition, they have not found any research that combines deep learning technology with spectrogram.

Spectrogram is a two-dimensional image that can reflect the essence of sound and can fully reflect the time-domain and frequency-domain information of sound [23]. The characteristics of spectrogram of different sounds are different, which is the premise of sound recognition using deep learning image processing method. There are differences in time-domain and frequency-domain information of different music types, which will be reflected in their spectrograms to a certain extent. This research combines deep learning with spectrogram and proposes a new music type recognition method. The feasibility of the method is verified by constructing the music spectrogram dataset and importing it into the deep learning model for training, so as to find a new and intelligent method for the research of national music recognition.

In this paper, from the perspective of multimodal data, music is decomposed into multidimensional data, and corresponding feature vectors are extracted for data fusion. At the same time, based on the depth confidence network, the classification of music is improved, that is, the fine-tuning node is added. The training set obtained from the fusion is trained in the improved deep confidence network, which can further improve the accuracy of music score classification. The main contributions are summarized as follows. (a) Simulate folk music of different spectrum, record corresponding music audio by Fourier transform and other methods under laboratory conditions, convert music audio into spectrum diagram, and obtain 2608 two-dimensional spectrum diagram images as datasets. Import the spectrum diagram dataset into the deep convolutional neural network GoogLeNet for music type recognition, with a test accuracy of 99.6%. (b) Parallel GoogLeNet technology based on inverse autoregressive flow is used. The unique improvement is that acoustic features can be quickly converted into corresponding speech time-domain waveforms, reaching the real-time level, improving the efficiency of model training and loading, and outputting more natural speech.

## 2. Design of the Classification System of the Spectrogram of the Folk Music

### 2.1. The Overall Framework Design of National Music Classification System

This system adopts MVC mode, which is popular in the industry, and develops the system based on B/S structure. It realizes the development goal of “high cohesion and low coupling,” separates page display, business logic, and data access, and is conducive to the hierarchical development of the system. The overall frame structure design of the system is shown in Figure 1. The user operates the system through the browser, and the operation request is transmitted from the view layer to the control layer through HTTP protocol. The control layer forwards these received requests to the business layer, which adopts different business logic to respond according to the different contents of user requests. After that, the response results are transferred to the view layer through the control layer and presented to the user in the form of HTTP pages.

Taking the user's classification request for opera as an example, the user submits the folk music information to be classified to the control layer through the view layer, and then the control layer transfers it to the business layer. After determining that the request is a classification request, the business layer calls the corresponding opera classification module to process it. After that, the classification results are transferred to the view layer through the control layer and displayed to the user at the specified position in the browser. Because the average power spectrum of the voice part of the music signal is affected by glottic excitation and oronasal radiation, it falls by 6 dB/octave in the high-frequency band above 800 Hz. In order to make the music signal obtain the spectrum with the same signal-to-noise ratio in the whole frequency band, it is necessary to strengthen the high-frequency part of the signal, which is the purpose of preemphasis processing on the signal. The spectrum can be made relatively flat by preemphasis processing, which is conducive to spectrum analysis and channel parameter analysis of the signal. The process of preemphasis is as follows: first, the music signal is digitized and then filtered by a preemphasis digital filter with 6 dB/octave high-frequency characteristics. In addition, the main goal of the development of this system is to realize a national music classification system, which can provide batch opera classification and annotation services for any user who has the needs of national music sorting and classification. This system selects the mel cepstrum coefficient that reflects the timbre and the pitch frequency, formant, and band energy distribution that reflect the melody. Combined with the deep confidence network model, it trains a large number of labeled samples to obtain the ability to classify national music and saves the classification model that meets the classification requirements through the test set to the system, so as to achieve the classification goal of unknown style national music. In addition, Chinese pronunciation has very complex prosodic rules, including whether the generated speech fully combines semantics with sound correspondence to express the real semantic relationship. The main function of the prosodic processing module is to label the text prosodically and process the prosodic features that can express the semantics such as the correct tone, stress, and tone of the language in the sentence.

### 2.2. System Hardware Design for Reorganization System

The main controller of the wireless distributed background music system is composed of core modules and functional modules. The hardware structure is shown in Figure 2. The core module adopts X4412CV2 as the core board, and the functional modules mainly include power circuit module, SD card and USB module, audio module, WiFi module, human-computer interaction module, and so on. The LCD screen in the human-computer interaction module adopts 7-inch TFT LCD screen, which supports backlight brightness adjustment.

The core module of this design uses Chuangzhan x4412cv2 core board as the development platform, which is a core board with low power consumption, high performance, and strong scalability. Exynos 4412 with Samsung cortex-a9 architecture is used as the main processor, and the running speed is as high as 1.5 GHz. It supports EMMC of various brands and capacities, uses dual-channel DDR3 design, has power sleep wake-up function, supports Android, Linux, and Ubuntu operating systems, and supports wired Ethernet expansion. The size of the core board is only 55 mm *∗* 55 mm. Furthermore, in this system, the reception and transmission of audio data are mainly completed through the WiFi module. In embedded systems, there are many kinds of WiFi interfaces, including SPI, SDIO, and USB. Based on the analysis of comprehensive performance, this design adopts the mt6620 chip of WiFi module MTK and uses the SDIO interface type as the connection type between WiFi module and x4412 board.

## 3. Research on the Classification Algorithm of National Music Rhythm Spectrogram Based on Biological Neural Network

### 3.1. Overall Structure Design of Classification Algorithm

Using vector sequence to represent the characteristic information of some aspects of music signal is called feature extraction. The performance of music classification system can be improved only by reasonably selecting the characteristic parameters of music signals. The overall framework diagram design of the algorithm is shown in Figure 3.

As shown in Figure 3, the classification of music rhythm mainly includes the following parts: (1) the determination of music rhythm category; (2) feature extraction of music clips; (3) training of music spectrum classification model; and (4) classification of the test set using the generated model. The main research content of this paper will also be structured according to these modules. In most content-based music classification systems, music content refers to the characteristic parameters of music itself. Therefore, for a classification system, the feature extraction of music signal is particularly important. This paper divides music features into three parts: bottom features, middle features, and advanced tags. The underlying music features can be sub-divided into timbre features and timing features. Timbre features are the most basic sound elements. Different sound sources produce different sound harmonics, and their timbre features are also very different. Experiments show that using timbre features can better reflect the music characteristics of the sound source, and it is easier to extract timbre features. Therefore, timbre features are usually selected as a parameter to reflect the music characteristics. Commonly used timbre feature parameters include SR, SC, and MFCC. The middle-level music features are based on the bottom-level music features, which reflect the melody, pitch, chord, and other characteristics of music. Prosody feature is another important parameter of music feature extraction, in which a large part of important information in music signal is included. Melodic features can be sub-divided into pitch, frequency, amplitude, pronunciation duration, rhythm, and so on. High-level labels can be divided into music emotion, music genre, etc. It is different from the basic and intermediate characteristics of music. The content of this part is usually not directly available, and the problem that it cannot directly correspond to the music signal is called the semantic gap problem. The purpose of extracting music signal features is to abstract the high-level label information of people on this music signal through these signal features.

In order to ensure sufficient model representation space and improve the recognition effect of the model, the basic prediction unit in this paper is audio segment, that is, it does not use full length music samples for prediction but uses short audio segments with a certain length for prediction. The model predicts each audio segment during training and prediction and takes the average value of the prediction results as the prediction result of the whole training sample. This method not only greatly reduces the requirement for input size but also enables the model to focus more on the capture of local features.

The general music classification system only selects one of these features as the music feature parameter. Although it also contains some music feature information, it will inevitably have some shortcomings, such as monotonous music information form, incomplete information content, and so on, which will affect the subsequent classification accuracy. This paper adopts the method of combining multiple features to extract the timbre features of the underlying music and the melody features (pitch frequency, formant, and band energy) of the middle-level music features from the original songs and then introduces the training set composed of these features to improve the accuracy of the classification system. The extraction of these two types of features is the integration of feature parameters extracted from music signals in time domain and frequency domain.

CNN deep neural network mainly combines generative pretraining and discriminant methods to process DBN, which is used to classify tasks and change all weights, which can improve the performance of the music classifications. The principle of discriminant scheme is as follows. Based on the existing network, attach a layer of nodes at the last layer, so as to achieve the purpose of fine-tuning.

### 3.2. Feature Extraction of Music Spectrogram

Audio signals convey linguistic and nonlinguistic information. The former refers to the semantic expression content delivered by the speaker, while the latter refers to the acoustic changes produced by the vocal system while the speaker completes the semantic expression. The two levels of information conveyed by voice and audio signals play a certain role in human emotional expression. In this paper, the audio of folk music is converted into corresponding spectrograms to construct datasets. Spectrogram is a two-dimensional image with color or gray changes that can fully reflect the essence of sound. The flowchart of music feature extraction is shown in Figure 4.

Spectrogram can reflect the time-domain information and frequency-domain information of sound at the same time, and it is highly intuitive. There are certain differences in the characteristics of spectrogram of different sounds. Convert audio into spectrogram, and the parameters used in the function are as follows: sampling frequency *f*_s_, overlap length (*L*_0_), Hamming window of Fourier transform (*w*), and number of points of Fourier transform *n*. Establish the short-time Fourier transform function of input signal *x*:

(1) $$\begin{array}{c} \text{specgram}\left(x\left(:\text{,}1\right),N,f_{s},w,L_{0}\right)\text{.} \end{array}$$

Taking time as the horizontal axis, the size *k* of the horizontal axis data is calculated by using the dimension *N*_*x*_of the input data, the Hamming window length *l*(*w*)during Fourier transform, and the window overlap length (*L*_0_):

(2) $$\begin{array}{c} k=\frac{\text{fix}\left(N_{x}-L_{0}\right)}{l\left(w\right)-L_{0}}\text{.} \end{array}$$

Taking frequency as the vertical axis, the magnitude of frequency *t* is determined by the number of points *N* of Fourier transform:

(3) $$\begin{array}{c} t=\left\{\begin{array}{cc} \frac{N}{2+1}\text{,} & N=\text{odd number},\\ \frac{\left(N+1\right)}{2}\text{,} & N=\text{even }number\text{.} \end{array}\right. \end{array}$$

In speech analysis, pitch generally refers to the sound produced by the vocal cord vibration when people pronounce voiced sound. When people pronounce unvoiced sound, because the vocal cord does not vibrate, it can be considered that this audio does not contain pitch. The pitch frequency is the reciprocal of the vocal cord vibration frequency when a person utters voiced sound. Fundamental frequency is widely used in speech analysis and synthesis and speech recognition. Especially, some researchers are also analyzing the relationship between pitch frequency and spectral prosody. Since intonation is a time function of the fundamental frequency of voice and intonation can reflect the emotional state of the speaker, the change of fundamental frequency is also closely related to the spectrum. Next, the effect of the fundamental frequency of the audio signal on the extraction of spectral features is analyzed from the mean, range, variance, and other aspects of the fundamental frequency trajectory. This paper selects the method of autocorrelation function detection to extract pitch frequency. The function *R*_*n*_(*k*) of signal *S*_*n*_ is defined as

(4) $$\begin{array}{c} R_{n}\left(k\right)=\overset{N-k-1}{\underset{m=0}{\sum }}S_{n}\left(m\right)S_{n}\left(m+k\right)\text{.} \end{array}$$

That is,

(5) $$\begin{array}{c} S_{n}\left(m\right)=s\left(m\right)w\left(n-m\right)\text{,} \end{array}$$

where *w*(*n* − *m*) is a window function.

### 3.3. Algorithm Design of Deep Neural Network

This paper designs the CNN structure figure as shown in Figure 5. Its core architecture includes nine inception modules. The classification algorithm reduces the number of channels through convolution, and computes after aggregating information. It effectively uses the computing power and obtains good classification performance while controlling the amount of computation and parameters. CNN can save parameters, speed up operations, and reduce overfitting The convolution and pooling operations of different scales are fused to fuse multidimensional features to further improve the recognition and classification effect. The network model of classification algorithm can fuse multiscale features and obtain good classification results. Therefore, this experiment applies it to this music classification task. Deep confidence network, abbreviated as DBN [14], is usually composed of multilayer RBW models, and the number of layers determines the accuracy of training, but it is also prone to overfitting. After a RBM is trained, the activation probability of its hidden unit will be used as the input data of the next RBM, in this order until all RBM models are trained. This training process is called generative pretraining. According to the data characteristics required for music emotion analysis, this paper improves the traditional DBN training method and adds the process of discrimination and fine-tuning on the basis of generative pretraining. The specific method is to add a node in each RBM hidden layer, improve the training accuracy of the whole model by fine-tuning the value of the ownership value, and provide labels of training data. The DBN model is composed of N layers of improved RBM, one layer of traditional RBM, and one layer of softmax. The first layer of RBM is the input layer of the DBN model and has *n* input vectors. Softmax layer is the output layer of DBN model, with *m* nodes representing *m* categories of music emotion.

LGC layer includes a set of predefined sparse Gabor filters, a nonlinear activation function, and a set of learnable linear weights. Due to the directional selectivity of Gabor, LGC layer can extract spatial texture features in all directions. LGC layer is actually composed of two convolution layers. The first layer performs convolution on the input image. Its convolution kernel is a set of fixed sparse Gabor kernels defined in advance, and the weight of this layer is fixed, which is not learnable in the process of training. The convoluted feature map is mapped by the nonlinear activation function, and the activation function used here is relu. In the second layer, the mapped features are linearly weighted to form the final feature map, which is used as the input of the next layer. This step consists of 1 × 1, and the weight of this layer can be learned in the process of training. Compared with the standard convolution layer, LGC layer has fewer learnable parameters with the same convolution kernel size and the same number of input and output channels. Suppose the number of channels of input data is *p*, the number of output channels is *Q*, and the size of convolution kernel is *n* × *m*. According to the convolution mechanism, the standard convolution layer requires *P* × *n* × *m* × *Q* learnable parameters, while the LGC layer requires *p* × *n* × *m* × *W* fixed parameters and *W* × *Q* learnable parameters, where *W* represents the channels of the middle layer and *w* × *Q* corresponds to a convolution kernel size of 1 × convolution operation of 1.

## 4. Experimental Results and Analysis

### 4.1. Data Source and Simulation Environment Settings

At present, there are several mature music datasets in the market, but most of these datasets only contain English tracks. Datasets specially built for Chinese traditional folk music are rare in the market. Therefore, to experiment with the classification model, we first need to build a folk music dataset. This paper uses web crawler tools to crawl music information and files from Chinese opera website, drama website, drama house, music, and other websites to the local way to build the database. Due to the size of the dataset, the MSD dataset itself does not provide original audio samples but provides audio feature data such as mel frequency cepstrum coefficient that has been calculated according to preset parameters, which does not conform to the experiment in this paper. Therefore, this paper uses the metadata provided by the MSD dataset to build a sub-dataset containing original audio samples.

The music clips used in this article are unified as 30 seconds, wav format, 16000 Hz sampling rate, mono. Because the first paragraph of the song has too much accompaniment, the last paragraph is almost less than 30 seconds. In this way, there are 6200 30 s music clips in total. At this time, the 3200 music clips generated are considered our preliminary music database because there may be duplicate clips for each music. By further deleting the duplicate clips of 6200 music clips, 4800 music clips are finally retained. The folk music files crawled from the network in this paper contain 4 types and 4800 tracks. Among them, there are 2600 songs and dance music, 800 kinds of rap music, 400 kinds of opera music, and 1000 kinds of instrumental music. After the selection of the music library is completed, each music segment will be manually calibrated next. Due to the subjectivity of emotional calibration of music, in order to enhance the credibility of the whole music library, the authors of this paper adopted the method of multiple people calibrating the same music segment.

In order to further verify the reliability of the experiment, the sonogram datasets were imported into the pretrained Resnet18 and Shufflenet for training. Resnet18 introduces the depth residual module to solve the gradient disappearance problem with the deepening of the network layers. After the convolution operation, a jump connection is added. When the accuracy decreases due to the deepening of the network layers, it can return to the shallow network to solve the gradient disappearance problem. Although Resnet18 has advantages in classification tasks by virtue of residual module, its network is relatively deep and its parameters are large. Shufflenet is one of the mainstream lightweight network models. The core operation of Shufflenet is to shuffle different channels, so as to give better play to the advantages of group convolution and further realize the balance between model lightweight and model performance improvement.

Software environment: using Python language, with the help of pycharm development environment and librosa speech extraction toolkit. The DBN model consists of *N* layers of RBM with fine-tuning nodes and one layer of unmodified RBM. Among them, the bottom input has 10 nodes, corresponding to 10 dimensional original data feature vectors. The number of cycles of pretraining is set to 100 times, and the number of fine-tuning cycles is set to 150 times. The top output layer has 5 nodes, corresponding to five types of folk music. Hardware configuration includes 16g memory, Intel Core i7-7700 processor, and NVIDIA 3050ti graphics card.

### 4.2. Convergence Verification of the Model

The system can test songs in two formats. Firstly, all songs under the whole testing folder are adopted, and finally count the number of classification errors of different categories of songs and the average accuracy of the classification of the last four categories of songs. The second test format can classify a music clip with unknown emotion category and get the category attribute of this music clip.

In this experiment, Resnet18 and Shufflenet are introduced into the music type recognition task to verify the reliability of the experiment, and the recognition effect of the model in this paper is compared with the large-scale model Resnet18 and the lightweight model Shufflenet. The data are imported into Resnet18 and Shufflenet, respectively, and the corresponding validation accuracy training chart, loss error training chart, and confusion matrix are obtained after the training of 20 epochs. Three network specific training parameters: the minimum batch is 64 times, the maximum iteration is 20 times, and the initial learning rate is 1 × 10^−4^, the verification frequency is 36 Hz, and the image input size is 224px × 224px.

The accuracy curve of validation accuracy training and validation is shown in Figures 6(a) and 6(b). The validation accuracy of thenetwork models in this paper, Resnet18 and Shufflenet, is 99.60% and 98.85%, both of which have high classification accuracy. The training process of the network model in this paper tends to be stable after the 20th epoch, and the accuracy of 99.60% is finally obtained, which shows that the method can effectively recognize music categories. Only two epochs are needed to improve the accuracy from 20% to 90%, which shows that the model has a high convergence rate. The model training accuracy curve tends to be consistent with the verification accuracy curve, and the loss rate loss tends to be close to 0 after the second epoch, which indicates that there is no fitting or underfitting phenomenon in the model training, which verifies the reliability of the experimental data. The simulation results in the above two cases (that is, the case of distinguishing the singer's gender and the case of not distinguishing the singer's gender) show that the performance of the GoogLeNet classification algorithm is better than that of the Shufflenet and Resnet classification algorithms. This is because the SVM method directly looks for an optimal hyperplane to distinguish the two categories of music and uses it as the final classifier. However, emotion classification of music itself has great fuzziness, and artificial emotion calibration of music has great subjectivity. The same music segment may be classified into different emotions. It is difficult to find a strong classifier with high classification accuracy directly for music emotion classification with large fuzziness, and the advantage of Resnet algorithm is to combine multiple weak classifiers to generate a strong classifier, which greatly improves the final classification performance. In order to verify the effectiveness of the two-tier classification system in this paper, the experimental results using the system structure in literature [18] and the system structure in this paper are compared, and it is found that the classification effect of the two-tier classification system structure in this paper is better.

In order to further verify the reliability and superiority, this paper classifies and verifies four types of folk music. Accuracy verification results of three network models are shown in Figure 7. The accuracy of GoogLeNet classification algorithm is significantly higher than that of Shufflenet, which also proves that the classification accuracy of finding a combination of multiple weak classifiers to form a strong classifier is significantly improved than that of finding a strong classifier alone. Of course, it is also a difficult task to distinguish them. The accuracy of this model is the highest whether using GoogLeNet algorithm or Shufflenet algorithm. For example, the first column of the confusion matrix indicates that 2480 samples are predicted as song types. From the data of confusion matrix, it can be calculated that the model test in this paper has achieved a high accuracy of 99.5%. Only 120 song type samples were mispredicted. The results show that this model has high accuracy in four categories: song, rap music, opera music, and instrumental music. Furthermore, in the process of training and verification, in order to ensure the consistency with the training parameters of GTZAN dataset, all samples with a time length of less than 30 seconds at the sampling frequency of 22050 Hz are eliminated in this paper. According to statistics, after the elimination according to the above rules, the original training set, development set, and evaluation set are eliminated by 5, 5, and 3 samples, respectively. In addition, other training details and training parameters are the same as those used in the GTZAN dataset. In the 5×10 fold cross-validation, the classification accuracy was the highest, reaching 87.68%, 5 × the average accuracy rate of 10-fold cross-validation is 87.11％. The number of national music classifications in the ISMIR2004 dataset is 5. The classification effect of Google network is better than that of Shufflenet and Resnet. This observation result is similar to that in the GTZAN dataset.

The sensitivity, specificity, accuracy, and other indicators of the test results of the three network models are shown in Table 1. By analyzing the model performance evaluation indicators such as sensitivity, specificity, and accuracy, it is found that the performance indicators of all models are above 97%, which indicates that the network model used in this experiment has good performance, which further verifies the accuracy of the network model in this paper.

## 5. Conclusion

With the development of various emerging art forms, the situation of traditional folk music is becoming increasingly severe. How to continue our unique traditional folk music is an urgent problem. This paper constructs a classification system of national music rhythm spectrogram based on biological neural network and uses classification technology to classify a large number of unorganized national music documents without labels, which will help national music better enter the vision of ordinary people to a certain extent. Firstly, the music information collected in the laboratory is converted into sound spectrum images, and the dataset containing 4800 sound spectrum images is obtained. Then, import the dataset into the deep convolution neural networks Resnet18 and Shufflenet proposed in this paper, and the test accuracy of 99.6%, 99.2%, and 99.2% is obtained. The experimental results show that the proposed network model has high recognition accuracy and can complete the classification of folk music. Music classification has important application value in multimedia applications. It shows that this method is reasonable and has better classification performance. The main reason is that there are fewer types of audio signal features, which limits the type resolution of music emotion. In the future, we will add other audio signal features and combination methods to the research of music emotion classification.

## Figures and Tables

**Figure 1:** System architecture design figure.

**Figure 2:** Schematic diagram of system hardware system.

**Figure 3:** Overall framework of the algorithm.

**Figure 4:** Flowchart of music feature extraction.

**Figure 5:** Structural design figure based on convolutional neural network.

**Figure 6:** Comparison of training results of the three models. (a) Accuracy. (b) Convergence error.

**Figure 7:** Accuracy verification of three network models.

**Table 1:** Model performance evaluation index.

Index	Our model			Resnet			Shufflenet		
	Sensitivity (%)	Specificity (%)	Accuracy (%)	Sensitivity (%)	Specificity (%)	Accuracy (%)	Sensitivity (%)	Specificity (%)	Accuracy(%)
Group 1	100	100	99.4	100	97.0	95.2	96.1	93.2	89.9
Group 2	100	100	99.6	99	96.0	95.1	94.3	92.4	88.7
Group 3	100	99.4	99.7	98	95.4	95.5	91.6	90.8	89.5
Group 4	99.3	99.5	99.4	96	95.0	95.3	90.4	89.7	90.0

## Data Availability

The data used to support the findings of this study are available from the corresponding author upon request.

## References

[1] Panganiban E. B., Paglinawan A. C., Chung W. Y., Paa G. L. (2021). SECG diagnostic support system (EDSS): a deep learning neural network based classification system for detecting ECG abnormal rhythms from a low-powered wearable biosensors. *Sensing and Bio-Sensing Research*.

[2] Castillo J. R., Flores M. J. (2021). Web-based music genre classification for timeline song visualization and analysis. *IEEE Access*.

[3] Liao Y. J., Wang W. C., Ruan S. J., Lee Y. H., Chen S. C. (2022). A music playback algorithm based on residual-inception blocks for music emotion classification and physiological information. *Sensors*.

[4] Tiple B., Patwardhan M. (2022). Multi-label emotion recognition from Indian classical music using gradient descent SNN model. *Multimedia Tools and Applications*.

[5] Khalifa Y., Mandic D., Sejdić E. (2021). A review of hidden markov models and recurrent neural networks for event detection and localization in biomedical signals. *Information Fusion*.

[6] Pati K. A., Gururani S., Lerch A. (2018). Assessment of student music performances using deep neural networks. *Applied Sciences*.

[7] Zhang K., Xu G., Han Z. (2020). Data augmentation for motor imagery signal classification based on a hybrid neural network. *Sensors*.

[8] Siphocly N. N. J., El-Horbaty E. S. M., Salem A. B. M. (2021). Top 10 artificial intelligence algorithms in computer music composition. *International Journal of Computing and Digital Systems*.

[9] Radha M., Fonseca P., Moreau A. (2019). Sleep stage classification from heart-rate variability using long short-term memory neural networks. *Scientific Reports*.

[10] Merchan F., Guerra A., Poveda H., Guzman H. M., Sanchez-Galan J. E. (2020). Bioacoustic classification of antillean manatee vocalization spectrograms using deep convolutional neural networks. *Applied Sciences*.

[11] Nag S., Basu M., Sanyal S., Banerjee A., Ghosh D. (2022). On the application of deep learning and multifractal techniques to classify emotions and instruments using Indian classical music. *Physica A: Statistical Mechanics and Its Applications*.

[12] Zhao K., Jiang H., Wang Z., Chen P., Zhu B., Duan X. (2020). Long-term bowel sound monitoring and segmentation by wearable devices and convolutional neural networks. *IEEE Transactions on Biomedical Circuits and Systems*.

[13] Hong S., Zhou Y., Shang J., Xiao C., Sun J. (2020). Opportunities and challenges of deep learning methods for electrocardiogram data: a systematic review. *Computers in Biology and Medicine*.

[14] Shah D., Narayanan A., Espinosa-Ramos J. I. (2022). Utilizing the neuronal behavior of spiking neurons to recognize music signals based on time coding features. *IEEE Access*.

[15] Fernandes M. S., Cordeiro W., Recamonde-Mendoza M. (2021). Detecting *Aedes aegypti* mosquitoes through audio classification with convolutional neural networks. *Computers in Biology and Medicine*.

[16] Ieracitano C., Mammone N., Bramanti A., Hussain A., Morabito F. C. (2019). A convolutional neural network approach for classification of dementia stages based on 2D-spectral representation of EEG recordings. *Neurocomputing*.

[17] Gauer J., Nagathil A., Eckel K., Belomestny D., Martin R. (2022). A versatile deep-neural-network-based music preprocessing and remixing scheme for cochlear implant listeners. *Journal of the Acoustical Society of America*.

[18] Korvel G., Treigys P., Kostek B. (2021). Highlighting interlanguage phoneme differences based on similarity matrices and convolutional neural network. *Journal of the Acoustical Society of America*.

[19] Ramírez J., Flores M. J. (2020). Machine learning for music genre: multifaceted review and experimentation with audioset. *Journal of Intelligent Information Systems*.

[20] Li J., Han L., Wang Y. (2022). Combined angular margin and cosine margin softmax loss for music classification based on spectrograms. *Neural Computing & Applications*.

[21] Tang H., Zhang Y., Zhang Q. (2022). The use of deep learning-based intelligent music signal identification and generation technology in national music teaching. *Frontiers in Psychology*.

[22] Liu C., Feng L., Liu G., Wang H., Liu S. (2021). Bottom-up broadcast neural network for music genre classification. *Multimedia Tools and Applications*.

[23] Ng W. W. Y., Zeng W., Wang T. (2020). Multi-level local feature coding fusion for music genre recognition. *IEEE Access*.

